# Research on Translation of Chinese Medicine Constitution (Tizhi) Academic Terms: Based on Memetics and Delphi Method

**DOI:** 10.1155/2022/2193459

**Published:** 2022-08-24

**Authors:** Siying Dong, Zixuan Zhao, Wenle Li, Yuyang Cai, Ziling Zhang, Minghua Bai, Ji Wang

**Affiliations:** ^1^Research Center of TCM Constitution and Reproductive Medicine, Beijing University of Chinese Medicine, Beijing 100029, China; ^2^School of Humanities and Foreign Languages, Hunan Agricultural University, Changsha 410128, China

## Abstract

**Background:**

With the continuous in-depth research of Chinese medicine constitution (tizhi) and the continuous expansion of cross research with new disciplines, internationalization will become the future trend of Chinese medicine constitution (tizhi). Translating the terms of Chinese medicine constitution (tizhi) into English is the first step for Chinese medicine constitution (tizhi) to go international. Language memes play an important role in information transmission in social interpersonal communication activities. The continuous replication and dissemination of translation memes make language spread and popularized. Because there is no fixed translation method at present, based on the particularity of Chinese medicine constitution (tizhi), we decided to use the Delphi method to complete the term translation research.

**Objective:**

The purpose of this study is to provide a standard and unified translation method for terms of traditional Chinese medicine (TCM) constitution with Chinese characteristics through the Delphi expert consultation strategy.

**Methods:**

Forward translation and expert consensus were conducted to complete this study. We sorted out the related terms of Chinese medicine constitution (tizhi) theory and invited an expert from the World Federation of Chinese Medicine Societies (WFCMS) to complete the initial forward translation. An expert of Chinese medicine constitution (tizhi) theory joined this process. Then, we invite relevant professionals to evaluate this translation version using the Delphi method.

**Results:**

Following a 3-round Delphi survey, the translation criteria of 61 (92.42%) terms were unified, and 5 terms resulted in no consensus and reached consensus on the translation method of Chinese medicine constitution (tizhi) theory. A major problem about how to translate “中医体质学” is identified. 25 experts participated in this study, and the drop-out rate is 0% in the 3-round Delphi survey. Translation challenges include the following: (1) translation methods of “Chinese medicine constitution (tizhi) theory”; (2) experts' understanding deviation on the definitions of some terms.

**Conclusions:**

The average mode, full score ratio, standard deviation, coefficient of variation, and variation ratio of expert scores are analyzed. The diversity of regions and professional titles of experts shows that they have a high degree of authority. The scores of terms indicate the consistent of study results, so they can be used as a reference for the translation of Chinese medicine constitution (tizhi) theory.

## 1. Introduction

In 1978, the research on Chinese medicine constitution (tizhi) (CMTZ) theory led by Wang Qi was put forward. This theory was based on the *Yellow Emperor's Internal Classic* and took *Treatise on Cold Pathogenic and Miscellaneous Diseases (Shanghan Zabing Lun)*, classic bibliography of TCM as the main theoretical and clinical guidance [1, 2], combined with many explorations and proofs in clinical and experimental studies. It is a theory that is mainly about human constitution characteristics, physiological and pathological characteristics of varying constitutions, analysis of reaction to disease, pathological nature and development trend, and guidance of disease prevention and treatment [3]. For the first time, it was confirmed that human's constitution is divided into nine types, from 2005 to 2007, and an epidemiological survey of 21948 people in nine provinces and cities of China was carried out, which confirmed the proportion of Chinese human's constitution [4]. Since 2009, the state administration of traditional Chinese medicine has added constitution (tizhi) identification to the standard of disease prevention and continuously expanded the scope of services in the next ten years [5]. CMTZ theory has been continuously developed and improved, forming a relatively complete theoretical system and becoming a characteristic project guiding the national health project of “preventive treatment of disease.”

Overseas, the influence of CMTZ theory is also expanding. The book *Systematic introduction to CMTZ* compiled by Wang Qi has been translated and published in the United States [6]. In addition, the Constitution of Chinese Medicine Questionnaire written by Wang Qi has also been translated into varying languages and applied in different countries [7]. With the continuous in-depth development of the research on CMTZ theory, some characteristic terms have been put forward, such as “three-differentiation clinical mode” and “treatment based on tizhi differentiation[8].” These terms are all newly created with unique expressions and definitions, which are different from any terms in TCM. As the carrier of TCM language, TCM terminology is an important part of linguistic research. Translating standardized terminology into local terms is an important step in the process of cross-cultural adaptation. At present, there is still no unified standard for the translation of TCM-related terms, but in the process of practice, we know that successful memes are easier to spread and replicate on the Internet [9].

Meme is “the information unit in the brain.” Professor He ZIran, who studies language application, believes that language meme plays an important role in information transmission in social interpersonal communication activities and is “the external and visual (auditory) expression of meme in the brain.” Memes in natural language are embodied in three aspects: education and knowledge transfer, the use of language itself, and communication and exchange through information [10]. Andrew Chesterman proposed that “the evolution of translation theory is caused by the continuous replication and dissemination of translation memes” [11]. At present, the research of memetics in China mainly involves the interdisciplinary research of memetics and translation, teaching, social language, and communication. A success meme should have three elements: “fecundity,” “longevity,” and “copying fidelity [9].”The translation methods of memetics are shown in Table 1.

Delphi method is often used in nursing practice [12], medical quality assessment [13], and translation [14]. Because we get feedback about translation through repeated surveys to obtain expert opinions, the opinions are usually unified after three rounds. As a team led by Academician Wang Qi, Research Center of CMTZ and Reproductive Medicine of Beijing University of Chinese Medicine, intends to sort out the Chinese version of CMTZ theory terms and translate them using memetics and Delphi method, it provides reference for domestic and foreign Tizhi theory researchers and promotes the popularization of CMTZ theory.

## 2. Methods

We first set up a steering group, which was responsible for drafting a detailed timetable, providing operational guidance, and facilitating the whole process. The steering group consists of a senior CMTZ theory expert, a methodological researcher, and two research secretaries. The flow chart of the whole study is shown in Figure 1.

### 2.1. Terminology Collection and Translation

All specialized vocabularies of CMTZ theory are sorted out, and the related concepts are listed in table. A total of 66 terms and their concepts were sorted out. The terminology comes mainly from the *Chinese Medicine Constitution (tizhi) theory* [15], which covers almost all terminologies and concepts of this area. In addition, there are also a few terms picked from recent papers, such as “Constitution (tizhi)-soil theory.” Those who involved in the translation work should meet a core set of qualification criteria, such as domain expertise and proficiency in the target language [16]. To make the translation more standardized and conform to the translation habits of TCM terms, we invited an expert from the Standards Department of the World Federation of Chinese Medicine Societies to cooperate with the experts in the steering group. Both experts have sufficient knowledge of TCM and English, and they will work together for preliminary translation. The main principles of translation refer to that of memetics preliminary forward translations of 66 terms which are shown in Table 2.

### 2.2. Identification of Core Issues

When preparing this questionnaire, the steering group invited some experts on CMTZ theory to discuss the key issue of this questionnaire, that is, how to translate “体质,” by brainstorming and referring to published documents or textbooks. We use PubMed to systematically search the literature about the tizhi theory from the establishment of the database to December 31^st^ 2020. As a result, by December 31^st^ 2020, among the 84 English literature related to the tizhi theory, there were 78 that used the term “中医体质学,” among which 52 (66.67%) used “(traditional) Chinese medicine constitution (constitution of/in (traditional) Chinese medicine),” 10 (12.82%) used “(traditional) Chinese medicine body constitution (body constitution of/in (traditional) Chinese medicine,” 6 (7.69%) used “body constitution,” and 5 (6.41%) used “constitution.” Other translations include “The constitutionology of Chinese medicine,” “The Chinese constitutional theory,” “TCM Physique,” “constitutional theory in Chinese medicine,” and “constitutional theory in Chinese medicine.” Specific search steps are shown in Table 3.

Based on the above results, we did a survey on whether to accept the word “tizhi” instead of “constitution.” A multiple-choice question was set at the beginning of the questionnaire. The question is set as “in order to meet the new situation of internationalization of TCM terms, after consulting experts on a small scale, it is considered that the translation of the word “体质” as “constitution,” which was used more in the past, is easy to cause ambiguity and cannot reflect the characteristics of TCM.” Therefore, we plan to change the English expression of the word into “Chinese medicine tizhi” in this standardized translation work. It is expected to provide a transition for popularizing the expression of Chinese traditional medicine characteristics. There are three options: agree, disagree, and others. After each option, experts are allowed to make their own suggestions freely. Finally, a questionnaire containing one multiple-choice question and 66 semistructured questions was generated.

### 2.3. Establishing Expert Database

As the CMTZ theory is a branch of TCM, and the research involves the application of CMTZ theory terms in English background, therefore, we mainly invited experts who knew the relevant background in the early stage of establishing the expert database. We mainly considered their literature contributions in this field and our personal contacts. We additionally invited 5 experts from the English language specialty of TCM. A total of 30 experts received the invitation letter. The letter briefly outlines the background, objectives, and expected number of rounds of the project, and the first-round questionnaire was attached. If experts agree to participate, the results would be returned directly by mail.

### 2.4. Delphi Expert Consultation

Experts reply by e-mail or fill them on an online questionnaire website (https://ww.wjx.cn/). We first collect personal information of participating experts, including gender, technical title, employer, occupation, major and years of professional experience, etc., which are used to analyze the authority of experts in statistics. Before each round of the survey, we will introduce our research purpose and details, as well as the inconsistent results of the previous rounds and answer part questions raised by experts. For experts' better understanding of the meaning of the terms and make accurate and objective judgments, each term in the questionnaire will be accompanied by its concepts, as long as these concepts can be found during collection. When the term is difficult to understand and the concept cannot be found, we will consult the opinions of CMTZ experts, and an explanation that is easy to understand will be attached to the term.

In the first round, one translation version will be given to each term, and experts will give their scores; questionnaires used by the traditional Delphi method typically consist of 4–9 points [17]. In this research, a 4-option question was used to measure the experts' attitude toward each item. Experts should look at each translation version and use a scale ranging from score 1 (very dissatisfied) to 4 (very satisfied) to classify their degree of agreement [18]. After each term, there is a comment box used to collect the reasons of their choice and provide an opportunity for experts to share their suggestions, which will be presented and resolved in the second and third rounds. When experts choose “2” or “1,” they can also put forward their own translation strategies. The consistency among respondents should be ≥75% [19, 20], or another round of voting should be implemented to reach a higher degree of agreement or confirm that no consensus has been reached. Experts' suggestions collected in nonagreed terms will be displayed on the new round list as new options or explanations for another vote. In an iterative manner, the same process will be repeated in certain expert groups. To ensure an adequate response rate in each round, experts are required to leave their real names to make sure they finished the questionnaire. To minimize the workload of experts, terms with an agreement level less than 50% in the previous round will not be discussed in the next, and the votes should be no more than 3 rounds.

#### 2.4.1. Results of the First Round

In this round, the questionnaire contains a total of 66 terms with 66 translations. We unified the translation version of 32 terms. For the first multiple-choice question, 17 (68%) of the experts agreed to translate “中医体质学” into “Chinese medicine constitution (tizhi),” while 7 (28%) disagreed and 1 (4%) chose others, figuring out the term can be translated into “traditional Chinese medicine constitution” as transition. We adopted their opinion and added this question to the next round, adding opinions about translation to the questionnaire in the second round.

#### 2.4.2. Results of the Second Round

The second-round questionnaire contains 34 terms and 85 translations, and 20 items achieved consensus. For the first multiple-choice question, 20 (80%) of the experts chose “Chinese medicine constitution (tizhi),” 4 (16%) thought it could be transitioned as “traditional Chinese medicine constitution”; 1 (4%) chose others and recommended to meet reader needs. We added this option to the third round. This important issue was agreed on in this round since more than 75% of experts agreed to translate into “Chinese medicine constitution (tizhi).”

#### 2.4.3. Results of the Third Round

In this round, the questionnaire contains of 14 terms and 49 translations. The average number of translations with the highest agreement among the remaining 5 entries ranged from 2.56 to 2.8, and failure to agree or agree with each other requires further exploration in future applications. The score results of the five items of each translation are shown in Figure 2. The translation results, scores, and statistics for each entry are shown in Table 4.

## 3. Experts in the Expert Panel

We sent emails to a total of 30 experts in China, and 25 experts responded to our questionnaire; the questionnaire response rate reached 83.33%. The experts who fulfilled the 3-round Delphi survey were 25, and response rates are 100%. The background of the experts is shown in Table 5. These experts come from 14 different units in 9 regions of China, male experts account for 40%, and female experts account for 60%. There are 80% of experts with doctor's degrees and postdoctoral degrees and 80% of experts with senior professional titles. Most experts account for two or more in scientific research and teaching and clinical activities, and the proportion of experts engaged in scientific research reached 96%. More than 50% of the experts are postgraduate supervisors. Experts comes from 10 major categories, including CMTZ, integrated traditional Chinese and Western medicine, traditional Chinese medicine, traditional Chinese medicine English, nutrition, and acupuncture, which shows professional diversity. Three of them are the academic heirs of traditional Chinese medicine, and they also provide opinions on translation methods with traditional Chinese medicine characteristics. We searched the literature before issuing the questionnaire. All experts knew something about CMTZ or published at least one relevant paper.

## 4. Limitations

First of all, with the continuous development of CMTZ theory, the number of terms will continue to expand. If the old translation results are not updated in time, there will be no unified translation method for some terms with the increase of terms. Secondly, due to the disciplinary limitations of this study, most of the experts we selected come from Beijing University of Chinese Medicine and major in CMTZ or those who have studied in this major. When answering questionnaires, compared with experts and staff of English translation, there may be certain professional limitations. For example, most experts have published professional related papers, so there may be some fixed pattern of thinking in word expression. Thirdly, most of the experts major in Chinese medicine disciplines, so the words used in translation from Chinese into English are not rigorous enough. We invited some experts majoring in Chinese medicine English to fix this problem. Finally, as some experts of TCM English major have some misunderstandings about the concept of CMTZ; in the latter round, we used simpler and understandable words to explain the terms with the premise of consulting the group experts. In the future, with the development of CMTZ, the terminology can be improved by more experts, and the results we deliver now do not necessarily represent the final version.

## 5. Discussion

Likert 5 and 7 scales are most used when using Delphi methods while few use Likert 4 scales [21]. When the consensus of the three scales is defined at 75%, it indicates that Likert scores should be ≥4/5 in Likert 5 scale and ≥6/7 in Likert 7 scale, while in Likert 4 scale, Likert scores should be ≥3. Unlike Likert 5, 7, and 9, Likert 4 has no median, so experts can only choose “agree” or “disagree” when scoring. However, as our questions are all semiopen, experts can raise their own opinions in fill-in questions whether they are satisfied with the translation results. If their opinions are neutral, they can state their position in the following table. The results show that most experts will choose a low score (most will choose (2) to promote the next round of discussion when they think the translation results are open to discussion).

In recent years, the CMTZ theory has been widely welcomed by scholars at home and abroad, and the number of related papers published has increased yearly. Translating its terms into English is conducive to global promotion. In this study, we invited experts from various regions, employers, genders, levels, and occupations in China and took three rounds of investigation based on the Delphi method. Experts are authoritative and the result was good and representative. It can be used as a preliminary reference for the translation of CMTZ terms, which will be convenient for later experts to unify the vocabulary when writing or to unify search terms when searching papers. This translation is based on the memetics and Delphi method, which is short in words and easy to understand, and provides a standardized method for other English-speaking countries. This is the first experiment to combine the translation of CMTZ terms with the Delphi method. Translating “中医体质学” into “Chinese medicine constitution (tizhi)” can better reflect the characteristics of TCMZ theory and provide a transition for the application of “tizhi.”

## Figures and Tables

**Figure 1:** Work-flow diagram of translation of the Chinese medicine (Tizhi) term.

**Figure 2:** Expert scoring of the 5 items in the Delphi inconsensus survey.

**Table 1:** The translation methods of memetics.

Essential factor	Explanation
Copying fidelity	The more faithful the copy is to the original, the higher the fidelity
Prolificacy	The faster and more memes are copied, the more they can spread. Industrial printing presses print more copies in a shorter time than manual printing presses.
Longevity	The longer the replication exists, the more stable the propagation is
Uniformity	The internal value of memes is consistent, which is not contradictory to the existing beliefs of individuals
Novelty	Memes can add new, unusual elements that can attract the attention of receptors
Simplicity	Memes should be easy to master and remember
Individual practicability	Memes should be able to help individuals achieve their personal goals
Significance	It should be easy to attract the attention of the receptor, for example, words loudly shouted or printed in the font of large posters
Expressive	Memes should be easily expressed in language or other forms of communication
Formality	The expression of memes is not easily changed by individuals or contexts
Infectivity	Individuals carrying memes should be willing to express, teach memes to others, or convert them into a belief
Conventionality	Memes can be supported by most individual ideas
Collective utility	Memes apply to groups rather than individuals

**Table 2:** Preliminary forward translations of 66 terms.

No.	Terminology	Translation in round 1
1	中医体质学说	Chinese medicine constitution (tizhi) theory
	ZHONG YI TI ZHI XUE SHUO	
2	中医体质分类法	Classification method of the Chinese medicine constitution (tizhi) theory
	ZHONG YI TI ZHI FEN LEI FA	
3	中医体质分类与判定标准	Criteria of Chinese medicine constitution (tizhi) classification and identification
	ZHONG YI TI ZHI FEN LEI YU PAN DING BIAO ZHUN	
4	中医体质量表	Chinese medicine constitution (tizhi) evaluation scale
	ZHONG YI TI ZHI LIANG BIAO	
5	九种体质	Nine constitutions
	JIU ZHONG TI ZHI	
6	平和质	Balanced constitution (tizhi)
	PING HE ZHI	
7	气虚质	Qi-deficiency constitution (tizhi)
	QI XU ZHI	
8	阳虚质	Yang-deficiency constitution (tizhi)
	YANG XU ZHI	
9	阴虚质	Yin-deficiency constitution (tizhi)
	YIN XU ZHI	
10	痰湿质	Phlegm-dampness constitution (tizhi)
	TAN SHI ZHI	
11	湿热质	Damp-heat constitution (tizhi)
	SHI RE ZHI	
12	血瘀质	Blood stasis constitution (tizhi)
	XUE YU ZHI	
13	气郁质	Qi-stagnation constitution (tizhi)
	QI YU ZHI	
14	特禀质	Special constitution (tizhi)
	TE BING ZHI	
15	过敏体质	Allergic constitution (tizhi)
	GUO MIN TI ZHI	
16	病理体质	Pathologic constitution (tizhi)
	BING LI TI ZHI	
17	兼夹体质	Compound constitution (tizhi)
	JIAN JIA TI ZHI	
18	偏颇体质	Unbalanced tizhi
	PIAN PO TI ZHI	
19	虚性体质	Deficient tizhi
	XU XING TI ZHI	
20	体质可分论	Constitution (tizhi) classifiable theory
	TI ZHI KE FEN LUN	
21	体病相关论	Constitution (tizhi)-disease correlation theory
	TI BING XIANG GUAN LUN	
22	体质可调论	Constitution (tizhi) regulating theory
	TI ZHI KE TIAO LUN	
23	禀赋遗传论	Natural endowment inheritance theory
	BING FU YI CHUAN LUN	
24	环境制约论	Environmental impact theory
	HUAN JING ZHI YUE LUN	
25	生命过程论	Life process theory
	SHENG MING GUO CHENG LUN	
26	形神构成论	Body-spirit composition theory
	XING SHEN GOU CHENG LUN	
27	肤体相关论	Constitution (tizhi)-skin correlation theory
	FU TI XIANG GUAN LUN	
28	体质土壤论	Constitution (tizhi) soil theory
	TI ZHI TU RANG LUN	
29	辨体	Constitution (tizhi) differentiation
	BIAN TI	
30	调体	Constitution (tizhi) regulation
	TIAO TI	
31	辨体-辨病-辨证	Constitution (tizhi)-disease syndrome differentiation
	BIAN TI-BIAN BING-BIAN ZHENG	
32	三辨模式	Three-differentiation clinical mode
	SAN BIAN MO SHI	
33	辨体论治	Treatment based on constitution (tizhi) differentiation
	BIAN TI LUN ZHI	
34	辨体施膳	Dietary therapy based on constitution (tizhi) differentiation
	BIAN TI SHI SHAN	
35	辨体养子	Child raising based on constitution (tizhi) differentiation
	BIAN TI YANG ZI	
36	辨体施护	Nursing based on constitution (tizhi) differentiation
	BIAN TI SHI HU	
37	辨体用方	Prescription based on constitution (tizhi) differentiation
	BIAN TI YONG FANG	
38	辨体质类型论治	Treatment based on constitution (tizhi) type
	BIAN TI ZHI LEI XING LUN ZHI	
39	辨体质状态论治	Treatment based on constitution (tizhi) condition
	BIAN TI ZHI ZHUANG TAI LUN ZHI	
40	三维中医体质模型	Three-dimensional Chinese medicine constitution (tizhi) models
	SAN WEI ZHONG YI TI ZHI MO XING	
41	胎传体质	Fetal infectious constitution (tizhi)
	TAI CHUAN TI ZHI	
42	体质保健	Health care based on constitution (tizhi)
	TI ZHI BAO JIAN	
43	体质辨识	Constitution (tizhi) identification
	TI ZHI BIAN SHI	
44	体质测评	Constitution (tizhi) assessment
	TI ZHI CE PING	
45	体质差异	Constitution (tizhi) difference
	TI ZHI CHA YI	
46	体质分型	Constitution (tizhi) classification
	TI ZHI FEN XING	
47	体质构成	Formation of constitution (tizhi) composition
	TI ZHI GOU CHENG	
48	体质类型	Constitution (tizhi) type
	TI ZHI LEI XING	
49	体质模型	Constitution (tizhi) model
	TI ZHI MO XING	
50	体质三级预防	Three-level prevention based on constitution (tizhi)
	TI ZHI SAN JI YU FANG	
51	体质三级预防体系	Three-level prevention system based on constitution (tizhi)
	TI ZHI SAN JI YU FANG	
52	体质三级预防学说	Three-level prevention theory of constitution (tizhi)
	TI ZHI SAN JI YU FANG XUE SHUO	
53	体质生理	Constitution (tizhi) physiology
	TI ZHI SHEGN LI	
54	体质现象	Constitution (tizhi) phenomenon
	TI ZHI XIAN XIANG	
55	体质研究	Constitution (tizhi) research
	TI ZHI YAN JIU	
56	体质演变	Constitution (tizhi) evolution
	TI ZHI YAN BIAN	
57	体质养生	Health maintenance based on constitution (tizhi)
	TI ZHI YANG SHENG	
58	体质预防	Disease prevention based on constitution (tizhi)
	TI ZHI YU FANG	
59	体质状态	Constitution (tizhi) condition
	TI ZHI ZHUANG TAI	
60	中医体质判定模型	Constitution (tizhi) identification model
	ZHONG YI TI ZHI PAN DING MO XING	
61	体质流行病学	Constitution (tizhi) epidemiology
	TI ZHI LIU XING BING XUE	
62	体质药理学	Constitution (tizhi) pharmacology
	TI ZHI YAO LI XUE	
63	体质遗传学	Constitution (tizhi) genetics
	TI ZHI YI CHUAN XUE	
64	体质表观遗传学	Constitution (tizhi) epigenetics
	TI ZHI BIAO GUAN YI CHUAN XUE	
65	体质代谢组学	Constitution (tizhi) metabolomics
	TI ZHI DAI XIE ZU XUE	
66	体质微生物学	Constitution (tizhi) microbiology
	TI ZHI WEI SHENG WU XUE	

**Table 3:** Search strategy used in PubMed.

No.	Search terms
1	constitution[Title/Abstract] OR physique[Title/Abstract]
2	Chinese medicine[All fields] OR traditional Chinese medicine[All fields]
3	1 and 2
4	Qi deficiency[Title/Abstract] OR Yang deficiency[Title/Abstract] OR Yin-deficiency[Title/Abstract] OR dampness[Title/Abstract] OR Damp heat[Title/Abstract] OR Phlegm[Title/Abstract] OR Blood stasis[Title/Abstract] OR Qi-stagnation[Title/Abstract] OR Allergic[Title/Abstract] OR special[Title/Abstract]
5	3 and 4

**Table 4:** Summary of the 66 items in the Delphi consensus survey.

No.	Terminology	Translation result	Delphi agreement	%	Average	Mode	Standard deviation	Coefficient of variation	Variation ratio
1	中医体质学说	Chinese medicine constitution (tizhi) theory	Round 2	75	3.00	3	0.85	0.28	0.60
	ZHONG YI TI ZHI XUE SHUO								
3	中医体质分类与判定标准	Criteria for classification and identification of Chinese medicine constitution (tizhi)	Round 3	75	3.00	3	0.80	0.27	0.52
	ZHONG YI TI ZHI FEN LEI YU PAN DING BIAO ZHUN								
4	中医体质量表ZHONG YI TI ZHI LIANG BIAO	Chinese medicine constitution (tizhi) scale	Round 3	75	3.00	3	0.75	0.25	0.56
5	九种体质	Nine types of constitution (tizhi)	Round 2	76	3.04	3	0.72	0.24	0.40
	JIU ZHONG TI ZHI								
6	平和质	Balanced constitution (tizhi)	Round 1	77	3.08	3	0.39	0.13	0.16
	PING HE ZHI								
7	气虚质	Qi-deficiency constitution (tizhi)	Round 1	77	3.08	3	0.39	0.13	0.16
	QI XU ZHI								
8	阳虚质	Yang-deficiency constitution (tizhi)	Round 1	77	3.08	3	0.39	0.13	0.16
	YANG XU ZHI								
9	阴虚质	Yin-deficiency constitution (tizhi)	Round 1	77	3.08	3	0.39	0.13	0.16
	YIN XU ZHI								
10	痰湿质	Phlegm-dampness constitution (tizhi)	Round 1	77	3.08	3	0.39	0.13	0.16
	TAN SHI ZHI								
11	湿热质	Damp-heat constitution (tizhi)	Round 3	79	3.16	3	0.61	0.19	0.40
	SHI RE ZHI								
12	血瘀质 XUE YU ZHI	Blood stasis constitution (tizhi)	Round 2	83	3.32	4	0.68	0.20	0.56
13	气郁质	Qi-stagnation constitution (tizhi)	Round 1	77	3.08	3	0.39	0.13	0.16
	QI YU ZHI								
14	特禀质	Special constitution (tizhi)	Round 1	77	3.08	3	0.39	0.13	0.16
	TE BING ZHI								
15	过敏体质	Allergic constitution (tizhi)	Round 1	78	3.12	3	0.32	0.10	0.12
	GUO MIN TI ZHI								
16	病理体质	Pathologic constitution (tizhi)	Round 2	78	3.12	3	0.77	0.25	0.60
	BING LI TI ZHI								
18	偏颇体质	Unbalanced constitution (tizhi)	Round 2	78	3.12	3	0.65	0.21	0.44
	PIAN PO TI ZHI								
19	虚性体质	Deficient constitution (tizhi)	Round 2	77	3.08	3	0.69	0.22	0.48
	XU XING TI ZHI								
20	体质可分论	Chinese medicine constitution (tizhi) classifiable theory	Round 3	76	3.04	3	0.77	0.25	0.48
	TI ZHI KE FEN LUN								
21	体病相关论	Constitution (tizhi)-disease correlation theory	Round 2	77	3.08	3	0.80	0.26	0.52
	TI BING XIANG GUAN LUN								
23	禀赋遗传论	Natural inheritance theory	Round 3	75	3.00	3	0.69	0.23	0.36
	BING FU YI CHUAN LUN								
24	环境制约论	Environmental impact theory	Round 2	78	3.12	3	0.65	0.21	0.44
	HUAN JING ZHI YUE LUN								
25	生命过程论	Life process theory	Round 2	77	3.08	3	0.69	0.22	0.36
	SHENG MING GUO CHENG LUN								
26	形神构成论	Body-spirit composition theory	Round 3	77	3.08	3	0.69	0.22	0.36
	XING SHEN GOU CHENG LUN								
28	体质土壤论	Constitution (tizhi)-soil theory	Round 2	80	3.20	3	0.63	0.20	0.44
	TI ZHI TU RANG LUN								
29	辨体	Constitution (tizhi) differentiation	Round 1	75	3.00	3	0.49	0.16	0.24
	BIAN TI								
30	调体	Constitution (tizhi) regulating	Round 2	78	3.12	3	0.77	0.25	0.48
	TIAO TI								
31	辨体-辨病-辨证	Constitution (tizhi)-disease-syndrome differentiation	Round 2	78	3.12	3	0.77	0.25	0.48
	BIAN TI-BIAN BING-BIAN ZHENG								
32	三辨模式	Three-differentiation clinical mode	Round 1	76	3.04	3	0.34	0.11	0.12
	SAN BIAN MO SHI								
33	辨体论治	Treatment based on constitution (tizhi) differentiation	Round 1	76	3.04	3	0.45	0.15	0.20
	BIAN TI LUN ZHI								
34	辨体施膳	Dietary therapy based on constitution (tizhi) differentiation	Round 1	76	3.04	3	0.45	0.15	0.20
	BIAN TI SHI SHAN								
35	辨体养子	Children raising based on constitution (tizhi) differentiation	Round 1	75	3.00	3	0.49	0.16	0.24
	BIAN TI YANG ZI								
36	辨体施护	Nursing based on constitution (tizhi) differentiation	Round 1	76	3.04	3	0.45	0.15	0.20
	BIAN TI SHI HU								
37	辨体用方	Prescription based on constitution (tizhi) differentiation	Round 2	82	3.28	3	0.60	0.18	0.44
	BIAN TI YONG FANG								
38	辨体质类型论治	Treatment based on constitution (tizhi) type	Round 2	84	3.36	3	0.56	0.17	0.44
	BIAN TI ZHI LEI XING LUN ZHI								
39	辨体质状态论治	Treatment based on constitution (tizhi) condition	Round 2	76	3.04	3	0.53	0.17	0.28
	BIAN TI ZHI ZHUANG TAI LUN ZHI								
40	三维中医体质模型	Three-dimension Chinese medicine constitution (tizhi) models	Round 1	75	3.00	3	0.28	0.09	0.08
	SAN WEI ZHONG YI TI ZHI MO XING								
42	体质保健	Health care based on constitution (tizhi)	Round 2	83	3.32	3	0.55	0.16	0.40
	TI ZHI BAO JIAN								
43	体质辨识	Constitution (tizhi) identification	Round 3	75	3.00	3	0.49	0.16	0.24
	TI ZHI BIAN SHI								
44	体质测评	Constitution (tizhi) assessment	Round 2	82	3.28	3	0.45	0.14	0.28
	TI ZHI CE PING								
45	体质差异	Constitution (tizhi) difference	Round 1	76	3.04	3	0.45	0.15	0.20
	TI ZHI CHA YI								
46	体质分型	Constitution (tizhi) classification	Round 3	77	3.08	3	0.63	0.20	0.28
	TI ZHI FEN XING								
47	体质构成	Composition of constitution (tizhi)	Round 2	81	3.24	3	0.71	0.22	0.16
	TI ZHI GOU CHENG								
48	体质类型	Constitution (tizhi) types	Round 3	79	3.16	3	0.61	0.19	0.40
	TI ZHI LEI XING								
49	体质模型	Constitution (tizhi) model	Round 1	78	3.12	3	0.43	0.14	0.20
	TI ZHI MO XING								
50	体质三级预防	Three-level prevention based on constitution (tizhi)	Round 1	75	3.00	3	0.57	0.19	0.32
	TI ZHI SAN JI YU FANG								
51	体质三级预防体系	Three-level prevention system based on constitution (tizhi)	Round 1	75	3.00	3	0.57	0.19	0.32
	TI ZHI SAN JI YU FANG								
52	体质三级预防学说	Three-level prevention theory of constitution (tizhi)	Round 1	77	3.08	3	0.48	0.16	0.24
	TI ZHI SAN JI YU FANG XUE SHUO								
53	体质生理	Constitution (tizhi) physiology	Round 1	79	3.16	3	0.37	0.12	0.16
	TI ZHI SHEGN LI								
54	体质现象	Constitution (tizhi) characteristics	Round 1	79	3.16	3	0.37	0.12	0.16
	TI ZHI XIAN XIANG								
55	体质研究	Constitution (tizhi) research	Round 1	79	3.16	3	0.37	0.12	0.16
	TI ZHI YAN JIU								
56	体质演变	Evolution of constitution (tizhi)	Round 1	78	3.12	3	0.43	0.14	0.20
	TI ZHI YAN BIAN								
57	体质养生	Health maintenance based on constitution (tizhi)	Round 2	78	3.12	3	0.77	0.25	0.48
	TI ZHI YANG SHENG								
58	体质预防	Disease prevention based on constitution (tizhi)	Round 1	76	3.04	3	0.45	0.15	0.20
	TI ZHI YU FANG								
59	体质状态	Constitution (tizhi) condition	Round 1	78	3.12	3	0.32	0.10	0.12
	TI ZHI ZHUANG TAI								
60	中医体质判定模型	Constitution (tizhi) identification model	Round 2	75	3.00	3	0.80	0.27	0.52
	ZHONG YI TI ZHI PAN DING MO XING								
61	体质流行病学	Constitution (tizhi) epidemiology	Round 1	76	3.04	3	0.45	0.15	0.20
	TI ZHI LIU XING BING XUE								
62	体质药理学	Constitution (tizhi) pharmacology	Round 1	77	3.08	3	0.39	0.13	0.16
	TI ZHI YAO LI XUE								
63	体质遗传学	Constitution (tizhi) genetics	Round 1	76	3.04	3	0.45	0.15	0.20
	TI ZHI YI CHUAN XUE								
64	体质表观遗传学	Constitution (tizhi) epigenetics	Round 1	76	3.04	3	0.45	0.15	0.20
	TI ZHI BIAO GUAN YI CHUAN XUE								
65	体质代谢组学	Constitution (tizhi) metabolomics	Round 1	76	3.04	3	0.45	0.15	0.20
	TI ZHI DAI XIE ZU XUE								
66	体质微生物学	Constitution (tizhi) microbiology	Round 1	76	3.04	3	0.45	0.15	0.20
	TI ZHI WEI SHENG WU XUE								
2	中医体质分类法	None							
	ZHONG YI TI ZHI FEN LEI FA								
17	兼夹体质<	None							
	JIAN JIA TI ZHI								
22	体质可调论	None							
	TI ZHI KE TIAO LUN								
27	肤体相关论	None							
	FU TI XIANG GUAN LUN								
41	胎传体质	None							
	TAI CHUAN TI ZHI								

**Table 5:** Characteristics of the participants.

Column		Number	%
Gender	Male	10	40.00
	Female	15	60.00

Highest education background	Bachelor's degree	2	8.00
	Master's degree	3	12.00
	Doctor's degree	20	80.00

Professional title	Primary title	1	4.00
	Intermediate title	4	16.00
	Deputy senior title	9	36.00
	Senior title	11	44.00

Nature of work	Scientific research work	24	96.00
	Clinical work	10	40.00
	Teaching	18	72.00

Major	Combination of TCM and Western medicine	8	32.00
	TCM	7	28.00
	TCM English	4	16.00
	Science of acupuncture and moxibustion	1	4.00
	Science of health maintenance of TCM	1	4.00
	Nutriology	1	4.00
	Epidemiology and medical statistics	1	4.00
	Smart healthcare	1	4.00
	Medical information engineering	1	4.00

Professional practical experience (years)	6∼10	10	40.00
	11∼20	7	28.00
	21∼30	4	16.00
	>30	4	16.00

Postgraduate supervisor	Ph.D. supervisor	7	28.00
	Master supervisor	6	24.00
	—	12	48.00

## Data Availability

The data used and/or analyzed during the study are available from the corresponding author on reasonable request.

## Abbreviations

CMTZ: Traditional Chinese medicine constitution (tizhi)
TCM: Traditional Chinese medicine.
